# Nursing Analysis Based on Medical Imaging Technology before and after Coronary Angiography in Cardiovascular Medicine

This article has been retracted.

**DOI:** 10.1155/2022/3279068

**Published:** 2022-04-15

**Authors:** Qin Li, Yangyang Yuan, Guangyu Song, Yonghua Liu

**Affiliations:** Department of Cardiovascular Medicine, Lianyungang First People's Hospital, Lianyungang, 222002 Jiangsu, China

## Abstract

With the advancement of technology, medical imaging technology has been greatly improved. This article mainly studies the nursing before and after coronary angiography in cardiovascular medicine based on medical imaging technology. This paper proposes a multimodal medical image fusion algorithm based on multiscale decomposition and convolution sparse representation. The algorithm first decomposes the preregistered source medical image by NSST, takes the subimages of different scales as training images, and optimizes the subdictionaries of different scales; then convolution and sparse the subimages on each scale encoding to obtain the sparse coefficients of different subimages; secondly, the combination of improved L1 norm and improved spatial frequency (novel sum-modified SF (NMSF)) is used for high-frequency subimage coefficients, and the fusion of low-frequency subimages improved the rule of combining the L1 norm and the regional energy; finally, the final fused image is obtained by inverse NSST of the fused low-frequency subband and high-frequency subband. Experimental analysis found that the bifurcation angle has nothing to do with the damage of the branch vessels after the main branch stent is placed. The bifurcation angle greater than 50° is an independent predictor of MACE after stent extrusion for bifurcation lesions. Experimental results show that the proposed method has good performance in contrast enhancement, detail extraction, and information retention, and it improves the quality of the fusion image.

## 1. Introduction

Medical imaging has completely changed the perception of health and disease for doctors and patients, enabling doctors to understand the internal conditions of the living body without having to dissect the body. In fact, if there is no medical imaging, it is impossible to form the field of modern medicine. Since medical imaging has become a routine examination method, the development of many breakthrough technologies, instruments, and equipment has led to tremendous changes in the field of medical imaging. With the rapid development of modern sensors and computer science and technology, medical imaging has gradually become an irreplaceable key component of clinical practical applications such as medical diagnosis, treatment planning, and surgical navigation. However, due to the diversity of imaging mechanisms, the information provided by different modes of medical images has its own limitations.

Due to the differences in imaging mechanisms of multimodal medical images, the tissue information reflected by them is also different, and a single-modal medical image cannot provide comprehensive and accurate information [1]. Therefore, it is of great significance to integrate medical image information of different modalities into one image to achieve information complementarity, facilitate medical diagnosis by doctors, and improve the accuracy of medical diagnosis [2]. This study provides a stepping stone for the advancement of coronary angiography in cardiovascular medicine.

The joint independent component analysis (jICA) model and the transposed independent vector analysis (tIVA) model are two effective solutions based on blind source separation (BSS). Blind source separation refers to the analysis of an unobserved original signal from multiple observed mixed signals. These solutions can fuse multiple models in a symmetrical and fully multivariate manner. Adali et al. apply these two models to the fusion of multimodal medical imaging data-functional magnetic resonance imaging (fMRI), structural MRI (sMRI), and electroencephalogram (EEG) data, which are derived from a cohort of healthy individuals and schizophrenia patients. They will show how the two models can be used to identify a set of components for all the methods used in the research, which collectively report the differences between the two groups. They discussed the importance of algorithm and order selection and the trade-offs to be made when choosing a model. Their method does not consider the possible impact of different data set testing [3]. In brain tumor surgery, tissue deformation during surgery (called brain shift) affects the quality and safety of the surgery. Brain shifts can move surgical targets and other important structures, such as blood vessels, thereby invalidating preoperative planning. Intraoperative ultrasound (iUS) is a convenient and economical imaging tool that can track brain shifts and tumor resections. Precise image registration technology based on iUS is a key but challenging technology to update preoperative MRI. The 2018 MICCAI Challenge (CuRIOUS2018) for correcting brain shifts through intraoperative ultrasound provides a public platform to benchmark the MRI-iUS registration algorithm on the newly released clinical data set. In this work, Xiao et al. showed the data, settings, evaluations, and results of 2018. It received 6 fully automated algorithms from leading academic and industrial research groups. All algorithms are first trained with a public resection database and then sorted according to the test data sets of 10 additional cases, which have the same data management and annotation protocol as the resection database [4]. Pinho et al. propose an extensible platform for multimodal medical image retrieval, which is integrated in open source PACS software with configuration file-based CBIR functions. They introduced in detail the technical methods to solve the problem by describing the main architecture of the problem and each subcomponent, as well as the available web interface and application multimode query technology. Finally, they use computational performance benchmarks to evaluate the implementation of the engine [5]. The data of these studies are not comprehensive, and the results of the studies are still open to question, so they cannot be recognized by the public and thus cannot be popularized and applied.

This paper uses the idea of metric learning to transform the classification problem of medical images into a measurement problem of similarity between medical image samples. Explore the effect of metric learning methods in the absence of medical image training data. The metric learning method is used to guide the feature extraction process of medical images, reduce the differences between individual clinical data, and overcome the problem of insufficient sample size.

The innovation of this paper is that:

1. this paper proposes a multimodal medical image fusion algorithm based on multiscale decomposition and convolutional sparse representation
2. this paper proposes a gating technology based on optical flow method to track biomarkers in vivo and automatically label respiratory nodules EE and EI

### 1.1. Medical Imaging Data Visualization Technology

#### 1.1.1. Medical Imaging Technology

*(1) Image Feature Extraction*. In terms of natural image processing and recognition, traditional image recognition methods usually design different feature extraction methods according to different objectives and targets [6]. Commonly used image feature extraction methods include image gray-scale features, such as overall or partial image mean, variance, kurtosis, and skewness. The calculation formulas are as follows:

The overall or local mean:

(1) $$\begin{array}{c} u=\frac{1}{N}\overset{N-1}{\underset{i=0}{\sum }}I\left(i\right). \end{array}$$

Image variance:

(2) $$\begin{array}{c} S^{2}=\frac{1}{N}\overset{N-1}{\underset{i=0}{\sum }}{\left(I\left(i\right)-u\right)}^{2}. \end{array}$$

Skewness of image:

(3) $$\begin{array}{c} Sk=\frac{N\sum_{i=0}^{N-1}{\left(I\left(i\right)-u\right)}^{4}}{\left(N-1\right)S^{4}}. \end{array}$$

Image kurtosis:

(4) $$\begin{array}{c} Ku=\frac{\sum_{i=0}^{N-1}{\left(I\left(i\right)-u\right)}^{4}}{\left(N-1\right)S^{4}}. \end{array}$$

*(2) Feature Dimensionality Reduction Method*. However, most of the above feature extraction methods are for two-dimensional grayscale images, and general shallow machine learning classifiers are mostly for one-dimensional features [7]. Therefore, for medical images with multiple dimensions, it is particularly important to reduce the dimensionality of medical images [8]. The most commonly used feature dimensionality reduction method is principal component analysis (PCA). PCA is a feature dimensionality reduction method for one-dimensional vector features [9]. For high-dimensional features, the commonly used method is to expand the high-dimensional data.

Feature dimensionality reduction is a very critical link in feature engineering. Successfully compressing high-dimensional features into the most representative low-dimensional features and then sending them to the machine learning model will greatly help the establishment of high-precision classifiers [10]. In the field of imagingomics, the more popular feature dimensionality reduction methods are LASSO method, principal component analysis, maximum correlation minimum redundancy mPMR, model dimensionality reduction method, statistical dimensionality reduction method, integrated dimensionality reduction law, etc. [11].

The PCA dimensionality reduction method is widely used in feature engineering in other fields and has good results, but it is relatively less frequently used in imaging omics [12]. PCA dimensionality reduction does not require the label information of the data. Its principle is based on the fact that the contribution of high-variance features in the total features is better than that of low-variance features. By building a sample matrix of the original data and features, the covariance matrix is calculated and the eigenvalues and eigenvectors of the covariance matrix are obtained. Several eigenvectors with higher eigenvalues are selected to form a new eigenmatrix according to requirements. Then, multiply the sample matrix and the new feature matrix to obtain the reduced dimensionality sample matrix; that is, the purpose of dimensionality reduction is achieved through coordinate mapping. The new low-dimensional features must be orthogonal to each other [13]. The advantage of PCA is that it can manually adjust the number of feature vectors to be selected and achieve different degrees of dimensionality reduction according to different needs [14]. The disadvantage of PCA lies in the inability to clarify the mapping relationship between the original imaging omics feature name and the research target, so it is impossible to intuitively explore the impact of the imaging omics feature on the research results [15].

The dimensionality reduction ideas of LDC and PCA are similar but not absolutely the same. LDC can also transform the original data set into a new feature subspace with a lower dimension# compressing the data while keeping as much relevant information as possible. In the two-dimensional feature space, although the dimensionality reduction along the *y*-axis ensures the maximum variance, it cannot distinguish the two categories well, which is not a good linear decision. The dimensionality reduction along the *x*-axis can distinguish the two categories well, so it is a better linear decision [16].

### 1.2. Transfer Learning Methods

Since the 1990s, in order to reduce the dependence of training models on calibration samples, transfer learning has been introduced into machine learning algorithms, greatly increasing the application range of machine learning algorithms. Transfer learning emphasizes the transfer of knowledge between different but similar fields. Usually, traditional machine learning algorithms are mostly supervised learning algorithms [17]. First, a large number of calibration samples are required. When there are sufficient calibration samples as training samples to learn a classifier, secondly, training samples and test samples need to obey the same distribution before they can be used. The classifier predicts the label of the test sample [18]. However, in practical applications, it is more difficult to calibrate enough samples for each field, which requires a lot of manpower and material resources.

Transfer learning is a new method for solving two domains with similar distributions. One domain has enough calibration samples, and the other domain has few or no calibration samples. It is necessary to use domain knowledge with enough calibration samples to solve the problem of no or only learning tasks in a small number of calibration sample areas [19]. Transfer learning can use the knowledge learned in the domain of sufficient calibration samples to solve another problem in the domain without calibration samples, that is, use the learned knowledge to solve problems in different but related fields. According to different scenarios and tasks, the way of transfer learning is also different. The use of transfer learning has a certain relationship with the calibration data volume of the target field and the similarity of the source field and the target field and the data volume. This similarity is very common; for example, the body structure of different people is similar.

### 1.3. Surface Rendering Technology

Surface rendering is a form of expression in scientific data visualization. Surface rendering usually constructs a three-dimensional data field from two-dimensional slice data and then constructs surface features such as planes and contours in the two-dimensional image [20]. Geometric primitives, such as curved surfaces or triangular patches, ignore the internal characteristics in the data. This is due to the fact that such geometric primitives do not focus on the detection of internal structures. After that, some related algorithms are used to splice and fit these geometric primitives, together with certain illumination and texture characteristics, to obtain a realistic three-dimensional visualization surface. The surface rendering method is a three-dimensional volume data visualization method, which fits the obtained data surface information to draw and ignores the internal information of the data [21]. It is characterized by reconstructing the surface contours of objects observed by researchers. Since the acquired data is part of the entire volume data, the internal information is discarded and only the surface information is drawn [22]. Computer graphics polygon drawing technology is used, and the graphics hardware acceleration function is used. Therefore, the surface drawing speed is fast and suitable for drawing tissues with clear surface characteristics. The common methods of surface drawing are voxel-based and contour-based surface drawing.

The voxel-based surface rendering method is also called “isosurface” extraction method. It is a common visualization technology and is generally applied to the fields of medicine, meteorology, and geology. Visualization is the theory, method, and technology of using computer graphics and image processing technology to convert data into graphics or images and display them on the screen and then perform interactive processing. This method first extracts surface data from a large amount of data and draws an “isosurface.” The surface of the object is composed of many small triangles. The three-dimensional image is drawn by extracting these triangles from the volume data and stitching them together. The object voxel studied in this method is the smallest unit of operation, so it is called a voxel-based surface rendering method, and because voxels need to be used to draw the isosurface, it is also called the “isosurface extraction method.”

The contour-based surface rendering is also called slice-level reconstruction. The basic idea of this method is to extract the contours of two-dimensional slices or sequence slices of the surface of the region of interest and use a certain method to classify and integrate the contours. Through a series of operations, the contour lines of the same attribute are obtained and connected and fitted. Get the surface of the region of interest and draw the surface contour.

The contour-based surface drawing method has four main steps: first extract the contour of the plane, then correspond to the contour between the slices, and then perform contour stitching and surface fitting. The extracted plane contours are segmented according to the attribute differences between the object and the background [23], such as grayscale, and the contours of different layers are compared by quantitative comparison of the overlapping parts of the contours, or the contours can be described in a way to make judgments. The contours on different layers correspond. For contour splicing, the corresponding points of the contour can be determined through related algorithms. Usually, the active contour method is used. A certain number of control points are selected on one contour, and a corresponding number of active points are selected on another contour, and the same sequence number points are deformed by external forces such as interaction force and displacement to determine the corresponding points. After finding the corresponding point, the approximate surface shape of the object is formed by the triangular or quadrilateral surface. Finally, a better object surface is presented through surface fitting.

However, there are some problems with the contour-based surface drawing step. What is more prominent is that in the process of contour splicing, when the number of object contours between adjacent layers is not equal, there may be a bifurcation problem, but the local information generated by the bifurcation cannot be determined. It needs to pass the geometry and topology of the global object.

### 1.4. Multi-Image Omics Feature Fusion

Corresponding imageomics features can be extracted from image data of the same period, and by fusing the imageomics features of image data of different periods, there is a higher probability that a model with higher generalization ability or higher accuracy can be obtained. In the fusion of multi-imageomics features, it is often used to use two fusion methods: the imageomics features of different phases are separately reduced in dimensionality, and then, the feature fusion is performed together for modeling; the imageomics features of different phases are first fused and then modelled after dimensionality reduction.

Feature engineering is an important part of photoomics modeling. The first method is to perform feature reduction independently according to the characteristics of the image data of different periods, and then the features after the independent dimensionality reduction are combined to form a new feature matrix. The new feature matrix can be further reduced in dimension or directly sent to the machine learning model for modeling. At this time, the feature matrix is more concise and more significant than the original feature matrix. The advantage of this method is that it can effectively avoid the problem of incomplete dimensionality reduction caused by high-dimensional features; that is, a large number of interfering features after fusion may affect the effect of a certain dimensionality reduction algorithm. The disadvantage of this method is that by first reducing the dimensionality of a certain type of image data feature, although it is ensured that the reduced feature has a small contribution to the category, it may be reduced by the features and some of the other prospective data. The features are correlated; that is, the combined features have a high degree of contribution to the total classification, so it is easy to overlook the correlation between the two different imageomics features.

The second method is to first combine the imageomics features of different types of image data, then perform dimensionality reduction to obtain a new feature matrix, and then send it to the model. The advantage of this method is that it can consider the relevance of two different types of features. The disadvantage is that a large number of features will interfere with the dimensionality reduction algorithm, which may affect the feature performance after dimensionality reduction. This drawback can be solved more effectively through hierarchical dimensionality reduction or mRMR algorithm.

## 2. Nursing Experiment before and after Coronary Angiography in Cardiovascular Medicine

### 2.1. Information

A collection of 1074 inpatients in the cardiology department of our hospital from January 2010 to January 2018 includes 730 male patients, accounting for 68.0%%, with an average age of 59.87 ± 9.82 years, and 344 female patients, accounting for 32.0%, with an average age of 61.24 ± 7.31 years; the ages of the selected candidates ranged from 33 to 85 years, with an average age of 61.27 ± 9.34 years.

### 2.2. Method

Using DSA contrast machine, after puncture through radial artery or femoral artery, CAG examination was performed by Judkins method. The degree of coronary luminal stenosis confirmed by CAG is expressed by the diameter method.

According to the results of CAG, the included patients were divided into two groups, namely, CAG-negative group and CAG-positive group. According to the number of coronary artery diseased branches, they were divided into three groups: single-vessel disease group, double-vessel disease group, and multivessel disease group. According to whether the ECG has ST-T changes, they are divided into ECG-negative group and ECG-positive group.

Use DSA machine to perform coronary angiography on the patient. After local infiltration of 1% lidocaine, anesthetize the puncture site, use Seldinger's method to puncture the patient's femoral artery or radial artery, and insert a 5F/6F Johnson artery sheath. Guided by the J-guide wire, send the angiography catheter to the left coronary artery (LCA) and right coronary artery (RCA) for selective coronary angiography (using standard Judkins method), multiposition projection to observe the lesions of the coronary arteries, including left main stem (LM), left anterior descending branch (LAD), left circumflex branch (LCX), and right coronary artery (RCA). LAD and LCX use the front position, right head position, right foot position, front foot position, spider position, and left head position for projection. RCA uses the left front oblique position and the front head position. The degree of coronary artery stenosis is judged by the visual diameter method, that is, (the diameter of the normal blood vessel near the heart of the stenosis − the diameter of the blood vessel at the stenosis)/the diameter of the normal blood vessel × 100%, based on the left and right coronary artery trunks and their main branches ≥ 2 mm. Arterial stenosis ≥ 50% is positive; no stenosis or stenosis < 50% means that the coronary angiography is negative. The interpretation of the angiography results is done by 3 doctors who do not know the patient's Holter chart results, have received uniform training, and have interventional qualifications, and take the average value.

### 2.3. Statistical Analysis

SPSS 24.0 statistical analysis software was used for data analysis. Quantitative data that satisfies the normal distribution are represented by the mean ± standard deviation (), and the comparison between groups is by *t* test; the quantitative data that is skewed distribution is represented by the median (interquartile range), and the Wilcoxon rank-sum test was used for the comparison between groups. Qualitative data is expressed as a percentage, and the comparison between groups is tested by Fisher's exact probability method. Multivariate logistic regression analysis was performed on the factors affecting ST-T abnormalities in Holter electrocardiogram, and *P* < 0.05 indicated that the difference was statistically significant.

## 3. Nursing Analysis before and after Coronary Angiography in Cardiovascular Medicine

### 3.1. ROC Curve of MPI and ECG Methods

For the acquired DCE-MRI, T2WI, and T1WI in-phase images, since the voxels of MR images have higher gray levels than natural images, the numerical difference between voxels is very large, and there are some sparse abnormalities. Consider using the following formula to normalize the voxel gray value range to [0,1]. Due to the limitation of medical image data quality and data completeness, the data set is very small. To prevent the model from overfitting, transpose, rotate, and flip the ROI data of the training set and test set to increase the amount of data. Rotating 90° can increase the data volume of the original data set by 3 times; horizontal and vertical flip operations can increase the data volume of the original data set by 2 times. Therefore, after using the data expansion method, the number of data samples can be increased to 6 times. We conducted experiments on data analysis and differentiation of HCC on the acquired image data set (Table 1).

As shown in Figures 1 and 2, the training model gradually tends to converge, loss gradually tends to 0, and dice gradually tends to 1, indicating that the model has achieved better performance in the training phase. It can be seen that the higher DSC indicates that the overall segmentation balance is better, and the values of precision and recall are very close, indicating that the learning is more stable.

As shown in Table 2 and Figure 3, the U-Net baseline trained with the dice loss function has the worst performance, with higher accuracy and recall scores, indicating that learning is unstable. In contrast, the U-Net model trained by the new focal Tversky loss function shows an increase in DSC and a more balanced precision and recall score due to the weight *α* in the loss function being higher than *β*. Injecting an input pyramid into the model can significantly improve the DSC, indicating that when the class imbalance is high, it is easy to lose the features of small damage.

### 3.2. Predictors of Branch Occlusion

As shown in Table 3, after correction using a multivariate regression model, it was found that the diameter ratio of MV/SB and the branch TIMI blood flow classification were two of the important predictors. In addition, the bifurcation angle, the stenosis rate of the branch diameter before the main branch stent placement, and the left ventricular ejection fraction (LVEF) also have a predictive effect on branch occlusion. The preoperative diameter stenosis rate of the proximal and distal main branch vessels is not an independent predictor of branch occlusion events. In addition, the lesion length of the proximal main branch vessel, the distal main branch vessel, the core of the bifurcation lesion, and the branch vessel have no predictive effect on the main branch vessel occlusion event.

The influence of bifurcation angle on the incidence of branch occlusion in PCI has been controversial. Some previous small sample studies have shown that the angle of coronary bifurcation has predictive significance. The smaller the angle, the higher the probability of branch vessel damage, restenosis, and major adverse cardiac events. The bifurcation angle has nothing to do with the damage of the branch vessels after the main branch stent is placed. The bifurcation angle greater than 50° is an independent predictor of MACE after stent extrusion for bifurcation lesions. In this study, a larger bifurcation angle can predict the occurrence of branch occlusion after the main stent is placed. This conclusion can be explained as follows: first, branch blood vessels with a smaller bifurcation angle, the blood flow shunts into the branch vessels more smoothly, and a larger bifurcation angle may increase the pressure difference and blood flow resistance of the blood flow shunt, thus increasing the risk of branch vessel occlusion; another explanation is that the greater the bifurcation angle, the smaller the shear stress of the vessel wall, and the oscillating shear force index at the bifurcation significantly increases, thereby promoting plaque in the bifurcation area of proliferation.

Chest pain is a common chief complaint of patient visits by general practitioners in the community. At least 1% of patients come to see a doctor because of chest pain. Clinicians and patients are more concerned about this symptom, because some potentially serious underlying diseases, such as coronary heart disease, myocardial infarction, and aortic dissection, need to be determined or ruled out. Although patients diagnosed with coronary heart disease account for only 10% of patients who go to the hospital for chest pain, the use of certain medical resources to exclude the diagnosis of coronary heart disease still has important public health value. Obviously, the use of an efficient and convenient screening method is particularly important when evaluating these symptoms. With the development of modern technology, electrocardiogram, Holter, cardiac exercise stress test, coronary CT angiography, etc. can all play a certain role in the diagnosis of coronary heart disease. Clinicians can choose detection methods according to the specific conditions of patients.

Nevertheless, CAG is still the current standard detection method for coronary heart disease, but it cannot be used for routine screening of coronary heart disease due to its insufficient economy and high technical requirements for clinicians. It is generally believed that the change of ST-T in ECG is related to insufficient coronary blood supply, and it is easy to operate and has low professional requirements. Therefore, ECG is often used as the most common method for screening coronary heart disease. Holter's application can continuously monitor and record the changes of the patient's ECG for 24 hours or more and can capture the accompanying changes in the ECG at rest, activity, and mood changes, significantly improving the detection of occult coronary heart disease and arrhythmia However, it is often found clinically that some patients with symptoms such as heart palpitations and chest pain have ST-T changes in Holter, but further CAG examination is negative, indicating that Holter ST-T segment changes are not characteristic of myocardial ischemia. Clinical factors are correlated with ST-T changes in Holter in patients with no obvious coronary stenosis.

As shown in Figure 4, according to whether Holter has ST-T changes, a group comparison analysis was performed, and the results found that the two groups had statistics on women, hypertension patients, LAD, LVEF, drinking history ratio, smoking history ratio, blood potassium level, and HGB. However, according to the logistic results, LAD, LVEF, proportion of drinking history, proportion of smoking history, blood potassium level, and HGB are not the influencing factors of ST-T changes in Holter with negative coronary angiography, while women and hypertension are the risk factors for ST-T changes in patients with Holter. Previous studies have shown that left ventricular thickness, thyroid function, etc. are usually considered to cause ST-T changes, but there is no statistical difference between the two groups in this study; age, hyperglycemia, hyperlipidemia, etc. are caused by coronary atherosclerosis. In this study, they accounted for a certain proportion of ST-T normal group and ST-T changed group, and the difference was not statistically significant. Therefore, it can be inferred that the above factors are not Holter in patients with negative coronary angiography risk factors for ST-T changes.

## 4. Conclusions

Medical imaging and medical image analysis have become key technologies in medical high-tech applications and are an indispensable part of modern imaging systems, which have greatly promoted the development of clinical diagnosis. Since the existing chest MRI dynamic imaging technology cannot automatically provide accurate gating information for the collected images of TIS patients, this paper proposes a gating technology based on the optical flow method to track biomarkers in the body to automatically label the respiratory nodes EE and EI. This gating technology allows patients to breathe freely during the medical image acquisition process. It only requires simple manual interaction and can complete a large amount of data annotation in a short time.

In view of the serious energy loss and low contrast of the fused image in the traditional multiscale-based medical image fusion method and the fusion method based on sparse representation using the L1 norm maximum fusion rule, the space for multimodal image fusion caused for the problem of inconsistency; this article first applies NSST decomposition to the source image to obtain the low-frequency image and a series of high-frequency images of the source image, perform inverse NSST to obtain the fused image, further save the details and contour information of the image better, improve the quality of the fused image, and verify the effectiveness and advancement of the proposed method through experimental verification.

Aiming at the research of Internet-based medical image registration, the medical image registration segmentation system is used to register the liver tissue in the abdominal organs, and the registration method based on feature points is adopted. The professional knowledge of medical experts to manually select the most iconic and unique feature points of the liver was used as the input in the registration method. Finally, the registration results of the liver area were evaluated by observation and quantitative methods to evaluate the effect of the system on liver registration. Such a registration experiment breaking platform provides a reliable computer-aided tool for clinicians to analyze images of liver cancer patients. The group studied in this study is small, and the experimental data lacks authoritativeness. Therefore, it is recommended to increase the number of experimental subjects in subsequent research.

## Figures and Tables

**Figure 1:** ROC curve.

**Figure 2:** Network training error rate.

**Figure 3:** Comparison of U-Net and its improved network evaluation indicators.

**Figure 4:** Holter in patients with negative coronary angiography.

**Table 1:** Evaluation index result table.

Category	Test set
DSC	0.788
Recall	0.803
Precision	0.864

**Table 2:** U-Net and its improved network evaluation index comparison table.

Network name	DSC	Recall	Precision
U-Net+DL	0.623	0.550	0.559
U-Net+FTL	0.628	0.699	0.587
Attention-UNet	0.661	0.638	0.773
Dense-UNet	0.600	0.659	0.774
FPA-UNet	0.688	0.681	0.746
DPA-UNet	0.830	0.714	0.931

**Table 3:** Quantitative analysis of coronary angiography.

Variable	OR	95% CI	*P* value
MV/SB diameter ratio	7.69	1.63-38.79	0.01
Bifurcation angle	1.12	1.11-1.08	<0.01
SB diameter stenosis rate	1.08	1.06-1.12	<0.01
TIMI blood flow classification of SB	3.63	1.49-8.77	<0.01
Left ventricular ejection fraction	1.11	1.04-1.15	<0.01

## Data Availability

No data were used to support this study.
